RETRACTED

# MMP-13 is involved in oral cancer cell metastasis

**DOI:** 10.18632/oncotarget.7942

**Published:** 2016-03-06

**Authors:** Shun-Hong Huang, Ching-Hsuan Law, Ping-Hsueh Kuo, Ren-Yu Hu, Ching-Chieh Yang, Ting-Wen Chung, Ji-Min Li, Li-Hsun Lin, Yi-Chung Liu, En-Chi Liao, Yi-Ting Tsai, Yu-Shan Wei, Chi-Chen Lin, Chien-Wen Chang, Hsiu-Chuan Chou, Wen-Ching Wang, Margaret Dah-Tsyr Chang, Lu-Hai Wang, Hsing-Jien Kung, Hong-Lin Chan, Ping-Chiang Lyu

**Affiliations:** ^1^ Department of Medical Sciences and Institute of Bioinformatics and Structural Biology, National Tsing Hua University, Hsinchu, Taiwan; ^2^ Department of Medical Sciences and Institute of Molecular and Cellular Biology, National Tsing Hua University, Hsinchu, Taiwan; ^3^ Department of Radiation Oncology, Chi-Mei Medical Center, Tainan, Taiwan; ^4^ Institute of Biomedical Sciences, National Sun Yat-Sen University, Kaohsiung, Taiwan; ^5^ Institute of Biomedical Science, National Chung Hsing University, Taichung, Taiwan; ^6^ Institute of Biomedical Science and Rong Hsing Research Center for Translational Medicine, National Chung Hsing University, Taichung, Taiwan; ^7^ Department of Medical Research and Education, Taichung Veterans General Hospital, Taichung, Taiwan; ^8^ Division of Chest Medicine. Department of Internal Medicine, Changhua Christian Hospital, Changhua, Taiwan; ^9^ Department of Biomedical Engineering and Environmental Sciences, National Tsing Hua University, Taiwan; ^10^ Department of Applied Science, National Hsinchu University of Education, Hsinchu, Taiwan; ^11^ Institute of Molecular and Genomic Medicine, National Health Research Institutes, Miaoli County, Taiwan; ^12^ Institute of Population Sciences, National Health Research Institutes, Miaoli County, Taiwan

**Keywords:** ECM, EMT, IF, MMP-13, OSCC

## Abstract

The oral cancer cell line OC3-I5 with a highly invasive ability was selected and derived from an established OSCC line OC3. In this study, we demonstrated that matrix metalloproteinases protein MMP-13 was up-regulated in OC3-I5 than in OC3 cells. We also observed that expression of epithelial–mesenchymal transition (EMT) markers including Twist, p-Src, Snail1, SIP1, JAM-A, and vinculin were increased in OC3-I5 compared to OC3 cells, whereas E-cadherin expression was decreased in the OC3-I5 cells. Using siMMP-13 knockdown techniques, we showed that siMMP-13 not only reduced the invasion and migration, but also the adhesion abilities of oral cancer cells. In support of the role of MMP-13 in metastasis, we used MMP-13 expressing plasmid-transfected 293T cells to enhance MMP-13 expression in the OC3 cells, transplanting the MMP-13 over expressing OC3 cells into nude mice led to enhanced lung metastasis. In summary, our findings show that MMP-13 promotes invasion and metastasis in oral cancer cells, suggesting altered expression of MMP-13 may be utilized to impede the process of metastasis.

RETRACTED

## INTRODUCTION

Oral cancer occurring often in oral cavity belongs to head and neck cancer; tumors at these sites typically cause eating, drinking, and speech difficulties as well as facial malformation resulting from treatment. Patients with advanced-stage oral cancer post a heavy familial, social, and financial burden. In the epithelial–mesenchymal transition (EMT) process, epithelial cells lose not only their cell polarity, but also their cell–cell adhesion ability; subsequently, some epithelial cells acquire migratory and invasive properties and develop into mesenchymal stem cells. These multipotent stromal cells can further differentiate into various cell types [1–3]. Matrix metalloproteinases (MMPs) are zinc-dependent endopeptidases belonging to a larger family of proteases known as the metzincin superfamily. MMPs are also considered to play a major role in cell processes such as migration (adhesion and dispersion), differentiation, angiogenesis, apoptosis, host defense and cancer metastasis. Moreover, MMPs can degrade all types of extracellular matrix (ECM) protein. For instance, one of the MMP superfamilies, MMP-13, is involved in the cleavage of the cell surface receptor TNF-α and the release of ligands. TNF-α can stimulate the metastatic pathway by attracting metastatic factors to the cell surface [4]. Turnover, remodeling, and degradation are the 3 predominant processes involved in ECM proteolysis [5]. Turnover is the breakdown and replacement of a protein or protein complex, and the turnover speed of many ECM proteins is relatively slow. Briefly, remodeling can be described as ECM breakdown and clearance in tissues undergoing structural change. Degradation refers to the control of or excessive matrix destruction. MMP family members have the function of degrading the ECM in both normal physiological and diseased cells, such as metastatic cells [6]. The degradation of collagenous ECM by MMPs is essential for invading malignant cells and for tumor-associated blood angiogenesis. For instance, intestinal tumorigenesis decreases in mice without MMP-7, and MMP-2-deficient mice exhibit reduced angiogenesis and tumor progression. To mimic oral cancer cell metastasis, a Transwell^®^ invasion assay was used. Cell migration is the movement of cells from one compartment chamber to the other and is due to a chemical concentration difference between the two chambers. Furthermore, cell invasion is a type of cell migration that requires moving through the ECM to reach and invade the blood vessels. Matrix metallopeptidase-13 (MMP-13) belongs to the MMP superfamily and is also called collagenase 3. MMP-13 in mice plays a critical role in musculoskeletal development. Mouse MMP-13 is markedly upregulated in the stroma during tumor growth and the progression of breast cancer. In humans, MMP-13 is highly overexpressed in patients with rheumatoid arthritis, [7] osteoarthritis, [8] and lymph angiogenesis of multiple myeloma [9]. However, whether MMP-13 plays a similar role in oral cancer remains unknown. Furthermore, no study has examined the association between MMP-13 and oral squamous cell carcinoma (OSCC) [10]. Metastasis can be categorized into 2 major phases. The first phase involves leaving the original organ to invade a distant organ, and the second phase involves colonization and outgrowth of the metastasized cancer cells. Initially, primary tumor cells acquire an invasion phenotype and attempt to degrade the ECM and intravasate the circulatory system through the bloodstream or lymph for dissemination to distant organs. When primary tumor cells circulate in the blood, they display properties of anchorage-independent survival. After cancer cells arrive at distant organs, the cancer cells must be able to adapt to the new microenvironment, survive and initiate proliferation. By using oral cancer cells carrying an shRNA to inactivate the MMP-13 gene function, we addressed the role of MMP-13 in the development of tumor metastasis to the lung *in vivo*. We demonstrated that the development and metastasis of the oral cancer OC3 cells *in vivo* depends substantially on MMP-13 expression.

RETRACTED

## RESULTS

### MMP-13 expression in higher in OC3-I5 than in OC3

Metastasis is a phenomenon in invasive cancer cells, and the degradation of the ECM can facilitate the migration of cancer cells. Therefore, the degradation of collagenous ECM by MMPs is essential for the invasion of malignant cells and tumor-associated blood angiogenesis. Considering the role of the MMP superfamily in cell invasion, we compared the expression of MMP-13 between the oral cavity squamous cell carcinoma OC3 and the invasive ability-enhanced OC3-I5 cell lines. The primary immunoblotting results revealed a higher expression of MMP-13 in OC3-I5 than in OC3 (Figure 1), thus supporting our speculation that OC3I5 cells pertain a higher matrix degradation ability.

**Figure 1:** Expression of MMP-13 in oral cancer OC3 and metastasis-enhanced OC3-I5 and the knockdown efficiency of siMMP-13 (**A**) Thirty micrograms of protein samples were diluted in a Laemmli sample buffer and separated using 1D SDS-PAGE following standard procedures. Expression of the target protein MMP-13 was monitored by immunoblotting. (**B**) OC3 and OC3-I5 cells were transfected with 50 nM siMMP-13, and the knockdown efficiency of various siMMP-13 strains and combinations were examined by immunoblotting. None represented for the mock cells. The combination of Strains 1, 9, and 11 revealed the optimal knockdown efficiency; hence, this combination was selected for further investigation. The concentration of 50 nM was selected as the experimental condition. Alpha-tubulin was used as the loading control.

RETRACTED

### Knockdown efficiency of siMMP-13

MMPs can degrade all types of ECM proteins; however, no association has been reported between the role of MMP-13 in oral cancer metastasis. Therefore, we examined the function of MMP-13 in OC3-I5 cell invasion. The OC3-I5 cells with an enhanced invasive ability and higher MMP3 expression were selected from the parental OC3 cells by using a Transwell^®^ invasion assay kit, and thus we inferred that MMP-13 might be responsible at least in part for the higher invasion ability. To inquire about this possibility, we used siRNA knockdown as a tool for downregulating MMP-13, and examined the effect of MMP-13 knockdown on the invasion ability of OC3-I5. Three strains of synthetic siRNA against MMP-13 were obtained from Invitrogen. The sequences 5′-CCG AGG AGA AAC AAT GAT CTT-3′ (Strain 1), 5′-GCT CCG AGA AAT GCA GTC TTT-3′ (Strain 9), and 5′-CTG TCA ATG AGA GCA TAA TTT-3′ (Strain 11) were designed against MMP-13. Furthermore, the efficiency of MMP-13 down regulation by various siRNA strains combinations was examined by Western immunoblotting analysis. A combination of Strains 1, 9, and 11 and the working concentration of 50 nM were found to be effective in down regulating MMP23 and thus selected for further experimentation (Figure 1).

### siMMP-13 downregulated the invasion ability of oral cancer cells in transwell invasion and migration assays

The Transwell^®^ invasion assay kit was employed to examine the invasion ability. The assay revealed a significant decrease in the invasion ability of both OC3 and OC3-I5 cells transfected with siMMP-13 compared with the scramble siRNA-transfected controls (mock). After siMMP-13 knockdown, the transwell invasion and migration abilities of the OC3 and OC3-I5 cells decreased by 40% and 60%, respectively. These results indicate that MMP-13 plays an important role in the migration and invasion abilities of those oral cancer cells (Figure 2).

**Figure 2:** Transwell invasion ability, transwell migration ability, and the number of cell attachments in oral cancer cells transfected with or without siMMP-13 (**A**) OC3 and OC3-I5 cells were transfected with 50 nM siMMP-13 or scramble siRNA (mock). An equal number of cells (50 000 cells/insert) were seeded into the matrix-coated upper chamber of the insert with a serum-free media. After 18 h, the invaded cells were fixed, stained with crystal violet, and microscopically viewed. The crystal violet was dissolved in an ethanol/acetic acid solution and quantified. The mock was considered the negative control. Error bars denote the mean ± SEM (*n* = 3). *P < .05, **P < .01, and ***P < .001 (**B**) The cells were transfected with siMMP-13 and recovered after 24 h. Furthermore, 5 × 10^5^ cells/insert were seeded with a serum-free media into the upper chamber without Matrigel coating. After 18 h, the migratory cells were fixed, stained with crystal violet, and microscopically viewed. The crystal violet was dissolved in an ethanol/acetic acid solution and quantified. The mock was considered as the negative control. Error bars denote the mean ± SEM (*n* = 3). *P < .05, **P < .01, and ***P < .001 (**C**) Mock and MMP-13-knockdown cells were seeded in a 12-well dish for 8 h. Furthermore, 1 × 10^5^ cells/well were seeded at 0 h, and the cells were washed with 1X PBS after culturing for 8 h. The number of cells was calculated using Brand, Neubauer. Data are presented as the mean ± SD of 3 independent experiments. *P* < .05 was considered statistically significant for the controls.

RETRACTED

### SiMMP-13 knockdown downregulates the number of cell attachment after cell subculture

Mock and MMP-13-knockdown cells were seeded in a 12-well dish for testing the attachment efficiency. 1 × 10^5^ cell per well were seeded at 0 h, and the cells were washed with 1X PBS after 8 h of culturing. Approximately 85% of OC3-I5 cells were attached in comparison with the other 3 cell lines (OC3, OC3-siMMP-13 and OC3-I5-siMMP-13); in particular, the siMMP-13–knockdown of OC3-I5 revealed that only approximately 60% of the cells were attached. Therefore, we considered that actin dots play a crucial role in cell attachment and migration. (Figure 2).

### EMT markers expression reveals that MMP-13 participates in epithelial–mesenchymal transition

Since OC3-I5 cells displayed an enhanced metastatic ability and a higher MMP-13 expression, and EMT is considered to be the initial step of metastasis, we inferred that MMP-13 might play some role in EMT. Therefore, we performed immunoblotting experiments to examine the involvement of MMP-13 in the molecules affecting of EMT. Corresponding with the migration/invasion data shown above, the result revealed that the OC3-I5 cells transfected with siMMP-13 showed reduced phosphorylation levels of Src. Higher expression of the EMT-inducing transcription factors was observed in the OC3-I5 than in the siMMP-13-knockdown cells. After MMP-13 knockdown in the OC3 and OC3-I5 cells, the EMT related transcription factors including Snail, SIP and Twist, were downregulated (Figure 3).

RETRACTED

**Figure 3:** Effects of siMMP-13 knockdown on the EMT status in invasive oral cancer cells (**A**) Total cell lysates were prepared from untreated or siMMP-13-treated cells. The cell lysates were immunoblotted with antibodies against EMT transcription factors, Twist, p-Src, Snail1, SIP1, JAM-A, and vinculin. (**B**) Total cell lysates were prepared from untreated or siMMP-13-treated cells. The cell lysates were immunoblotted with antibodies against EMT downstream proteins, E-cadherin, and vimentin. Alpha-tubulin was considered the loading control. According to ImageQuant TL 1D gel analysis, after each value was normalized with its alpha-tubulin, the obtained values were normalized with their antibodies stained in OC3. (**C**) Antibodies used in the immunoblots are listed in the table.

### siMMP-13 can regulate downstream EMT markers and block E-cadherin expression

Transcription factors such as Snail1 and Slug1, which block E-cadherin, are considered EMT-promoting factors. Slug1 binds to E-cadherin promoter and represses its transcription. This decrease in E-cadherin is accompanied by an increase in the expression of mesenchymal-associated proteins, including vimentin. Immunoblotting revealed that the expression of E-cadherin, cellular structure, and cell–matrix interaction components JAM-A and vinculin were higher in the OC3 cells (Figure 3). By contrast, the expression of the EMT marker molecule vimentin was the higher in the OC3-I5 cells. In both OC3 and OC3-I5, MMP-13 knockdown resulted in down regulation of vimentin.

### Both OC3 and OC3-I5 cells exhibited motility defects after MMP-13 knockdown in wound-healing assays

Wound-healing assay provides a simple means for monitoring directional cell migration and *in vitro* interaction. OC3 and metastasis-enhanced OC3-I5 cells were transfected with a siMMP-13-knockdown vector, and 2 × 10^5^ cells per well were seeded onto a 12-well dish and incubated for 24 h (approximately 90% confluence). A linear wound was generated using a sterile 10-μL plastic pipette tip through a premarked line to assay for wound-healing; microscopic observations were recorded from 0 to 24 h after the wound scratching on the surface of a confluent cell layer. Wound healing was measured in the absence of a chemotactic gradient. Both the OC3 and OC3-I5 cells exhibited motility defects after MMP-13 knockdown in the wound-healing assays, as revealed by the small healing area observed under an optical microscope. Initially, the scratching surface was similar; after 24 h, OC3-I5 cells with a higher migratory ability displayed a significantly greater wound healing ability than the OC3 cells. The healing area was calculated using Axio Vision 4. After MMP-13 knockdown, the healing area of OC3–siMMP-13 decreased by approximately 32% compared with that of OC3; similarly, the healing area of OC3-I5–siMMP-13 decreased by approximately 29% compared with that of OC3-I5. (Figure 4) Data are presented as the mean ± SD of 3 independent experiments. *P* < .05 was considered statistically significant for the controls

**Figure 4:** After siMMP-13 knockdown, the wound-healing migration ability was downregulated in the oral cancer cells Mock and MMP-13 knockdown cells were seeded in a 12-well dish overnight. A wound was created at 0 h. (**A**) Photographs of the wound at 0, 8, 16, and 24 h. (**B**) Size of the healing area, which was calculated using Axio Vision 4. Error bars denote the mean ± SEM (*n* = 3). *P < .05 and **P < .01.

RETRACTED

### MMP-13 is essential for protein synthesis in oral cancer by staying in the G1 phase

The cell cycle involves a series of stages leading cell duplication into daughter cells. This cycle includes 4 phases: G1, S, G2, and M phases. The cells increase in size in the G1 phase, and the G1 checkpoint control mechanism ensures that conditions are feasible for DNA synthesis. During this phase, the biosynthetic activities of the cells occur at a high rate, and the increase in protein levels and the number of organelles, including the mitochondria and ribosomes, thus increase the cell size. During the G2 phase, the cells continue to grow. After the G2 checkpoint control mechanism is completed, the cells enter the M (mitosis) phase and divide [11–14]. After downregulation by siMMP-13, the G1 phase of the invasive OC3-I5 cell line decreased by approximately 18.9%. Furthermore, the S phase increased by approximately 3.3%, and the G2/M phase increased by approximately 16.4%. In the less invasive OC3 cell line, after downregulation by siMMP-13, the G1 phase decreased by approximately 19.9%, the S phase increased by approximately 3.7%, and the G2/M phase increased by approximately 11.2%. Overall, MMP-13 is essential for protein synthesis in oral cancer by promoting cell entry into the G2/M phase. Therefore, the decrease in MMP-13 knockdown cells in the G1 phase subsequently progresses to the S and G2/M phases. Accordingly, we speculate that MMP-13 is necessary for synthesizing protein and energy organelles in the G1 phase, thus providing energy for invasive cancer cells to degrade the ECM and translocate from the original location to distant colony regions. (Figure 5).

RETRACTED

**Figure 5:** Downregulation in the G1 phase is induced by siMMP-13 transfection in oral cancer cells Cells in various stages of the cell cycle after siMMP-13 knockdown, and MMP-13–silenced OC3 and OC3-I5 cells incubated with PI. After incubation for 15 min, the cells were analyzed through flow cytometry, and the DNA content was quantified. (**A**) The cell count is represented on the Y axis, and PI is represented on the X axis. Cell cycle status was analyzed according to the DNA content, and G_l_, S, and G_2_/M phases were calculated. The G1 phase was downregulated, and the S and G2/M phase were upregulated. (**B**) Percentage of the cell cycle status. Error bars denote the mean ± SEM (*n* = 3). *P < .05 and **P < .01.

### MMP-13 played a crucial role in focal adhesion formation

Because OC3-I5 cells have a faster migratory and thus likewise the wound healing ability, it can be inferred that they many actin dots inside the cell. Actin dots and the nucleus were stained with phalloidin and DAPI, respectively (Figure 6). After they were colocalized with these 2 dyes, the location of the actin dots in the cell was visualized by fluorescence microscopy. Fluorescence microscopy revealed the effect of MMP-13 knockdown on actin staining. Phalloidin staining revealed actin dots around the cell surface with or without MMP-13 knockdown in OC3 cells. The conditions in the OC3-I5 cell line were quite different. Numerous actin dots were distributed in the cells, and some significant and bright light was also observed at the cell surface and edges. Statistical data revealed that the quantity of actin dots in the OC3-I5 was approximately 8000, which was approximately 4-fold that observed in the siMMP-13-knockdown cells. The result indicated that MMP-13 played an important role in focal adhesion formation for the OC3-I5 cells.

**Figure 6:** Effect of oral cancer cells on focal adhesion formation in the treated siMMP-13 OC3 and OC3-I5 cells were transfected with siMMP-13 and recovered after 24 h. The cells were seeded on a 12-mm glass slide and incubated overnight. Subsequently, the cells were fixed and hybridized with phalloidin for 1 h and DAPI for 1 min. (**A**) Photographs of the actin dots. (**B**) Microscopic images showing the count and quantification of the actin dots. The mock was considered the negative control. Scale bar: 20 μm. Error bars denote the mean ± SEM (*n* = 3). *P < .05 and ***P < .001.

### Using MMP-13 plasmid-transfected 293T cells to enhance MMP-13 expression in the OC3 cell line

Lentivirus particles are produced from 293T cells through the transient transfection of MMP-13 plasmids that encode for virion components. The lentiviral supernatant can be produced by cotransfecting 293T cells, which is the liquid of the MMP-13 plasmid we used for infecting the oral cancer OC3 cell line. Immunoblotting ensured that the expression of the 293T cells and OC3 cell line infected with the MMP-13 plasmid was more than that of uninfected cell line. We used this MMP-13-overexpression cell line to determine whether MMP-13 is involved in oral cancer metastasis *in vivo*. (Figure 7).

RETRACTED

**Figure 7:** Using MMP-13 plasmid-transfected 293T cell to enhance MMP-13 expression in OC3 cancer cell line and the effect of shMMP-13 knockdown on the transwell migration and invasion ability of oral cancer cells (**A**) pLenti virus with MMP-13 plasmid-infected 293T cell for overexpressing virus with MMP-13. A large amount of the virus was transfected into the OC3 cells to stably express MMP-13. Cell lysates were immunoblotted with antibodies against MMP-13. Alpha-tubulin was considered the loading control. (**B**) Cells were transfected with shMMP-13 and recovered after 24 h. Furthermore, 5 × 10^5^ cells/insert were seeded in a serum-free media into the upper chamber without Matrigel coating. After 18 h, the migratory cells were fixed, stained with crystal violet, and microscopically viewed. The crystal violet was dissolved in an ethanol/acetic acid solution and quantified. The mock was considered the negative control. Error bars denote the mean ± SEM (*n* = 3). *P < .05, **P < .01, and ***P < .001 (**C**) OC3 and OC3-I5 cells were transfected with shMMP-13 or scramble shRNA (mock). An equal amount of cells (5 × 10^5^ cells/insert) was seeded into the matrix-coated upper chamber of the insert with serum-free media. After 18 h, the invaded cells were fixed, stained with crystal violet, and microscopically viewed. The crystal violet was dissolved in an ethanol/acetic acid solution and quantified. The mock was considered the negative control. Error bars denote the mean ± SEM (*n* = 3). *P < .05, **P < .01, and ***P < .001.

### shMMP-13 downregulated the migration ability of oral cancer cells in the transwell migration assay

The transwell migration assay revealed a significant reduction in the migration ability of both the OC3 and OC3-I5 cell lines transfected with shMMP-13 compared with the scramble shRNA-transfected controls (mock). After shMMP-13 knockdown, the transwell migration ability of the OC3 and OC3-I5 cells decreased by 50% and 76%, respectively. (Figure 7) These results also indicate that MMP-13 plays a critical role in migration ability. When the primary cancer cell degrades the ECM, they can colonize throughout the body, particularly in organs with a high quantity of capillary blood vessels, such as the lungs and kidneys. In transwell invasion and migration assays, the transwell membrane is a cell membrane simulator, and the aggressive cancer cell enhances the invasion ability because of the high expression of metastasis-related proteins such as MMP-13, a MMP superfamily member.

RETRACTED

### shMMP-13 downregulated the invasion ability of oral cancer cells in the transwell invasion assay

The transwell invasion ability assay revealed that the invasion ability of both OC3 and OC3-I5 cells transfected with shMMP-13 significantly decreased compared with the scrambled shRNA-transfected controls (mock). After shMMP-13 knockdown, the transwell invasion ability of the OC3 and OC3-I5 cells decreased by 50% and 70%, respectively. (Figure 7) These results indicate that long-term shMMP-13 can be used in animal tests.

### Downregulation in the G1 phase is induced by shMMP-13 transfection in oral cancer cells

The cells at a density of 10^6^ cells/mL were stained with and resuspended in PI dye at the concentration of 50 μg PI and 10 μg RNase per 1 mL of PBS, and were then incubated on ice in the dark for 20 min. We subsequently used flow cytometry (Accuri CFlow) to examine the emission of PI staining at 575 nm in order to analyze the percentages of cell cycle in the OC3 cells as well as the derivative OC3-I5 cell line that was screened using the transwell invasion assay (with or without MMP-13 shRNA knockdown). Data were further analyzed using CFlow Plus analysis software (BD Biosciences). We determined that the G1 phase decreased by 5.87% in the OC3 cells and by 0.7% in the derivative OC3-I5 cell line; the S phase increased by 0.5% in the OC3 cells and decreased by 0.2% in the derivative cell line OC3-I5. Furthermore, the G2/M phase increased by 2% in the OC3 cells and increased by 3.7% in the derivative OC3-I5 cell line after treatment with the MMP-13 shRNA-knockdown. (Figure 8) Thus, the MMP-13 knockdown had a direct G2 arrested effect on the OC3 and OC3-I5 cells. By contrast, we determined that the G1, S, and G2/M phases decreased by 5.9%, 0.2%, and 2.1%, respectively, in the OC3/MMP-13-overexpression cells. In the G2 arrest phenomenon, the G2/M DNA damage checkpoint retains the cell in the G2 phase before mitosis in response to genotoxic stress, such as UV radiation, oxidative stress, and DNA intercalating agents, in a p53-dependent or -independent manner. Moreover, DNA damage signals cause the activation of the transcription factor p53. Therefore, in the following test, we examined the increase in the volume of p53 and cyclin B1/CDK1 in the G2/M arrest by using immunoblotting.

**Figure 8:** Downregulation in the G1 phase was induced by shMMP-13 transfection in oral cancer cells MMP-13-silenced OC3 and OC3-I5 cells were incubated with PI for 15 min. Subsequently, the cells were analyzed through flow cytometry, and the DNA content was quantified. (**A**) Cell count is represented on the Y axis, and PI is represented on the X axis. Cell cycle status was analyzed according to the DNA content, and the G_l_, S, and G_2_/M phases were calculated. The G1 phase was downregulated, and S and G2/M phases were upregulated after shMMP-13 knockdown. The G1 and G2/M phases were downregulated, and the S phase was upregulated after MMP-13 overexpression. (**B**) The percentage of the cell cycle status was quantified. Error bars denote the mean ± SEM (*n* = 3). *P < .05 and **P < .01.

RETRACTED

### Stable knockdown of MMP-13 in human oral cancer cells decreases metastasis *in vivo*

The function of MMP-13 in oral cancer invasion, migration, and proliferation reamins unknown; therefore, we examined the role of MMP-13 in oral cancer invasion *in vivo*. The shMMP-13 plasmid DNA was transfected in the OC3 and OC3-I5 cells; stably knocked down cell lines were established using puromycin selection, which was performed every 2 passages until the cell viability was unaffected by puromycin. Five-week-old BALB/cAnN.Cg–Foxnlnu/CrlNarl female mice were housed in a specific-pathogen-free environment [15]. One week after housing, the mice were injected with human oral cancer cells. Furthemrore, 2 × 10^6^ OC3 and OC3-I5 cells stably transfected with shMMP-13 were washed with PBS and subcutaneously inoculated into the vein of the mice tails (6 per group). The mice were anaesthesized and sacrificed using CO_2_ 20 d after the implantation, and the lungs were removed and fixed in 10% formalin. The weight of the lungs was measured. The stable knockdown of MMP-13 in the human oral cancer cells decreased the metastasis, and the overexpression of MMP-13 in the less-invasive OC3 cell line increased the *in vivo* metastasis. According to the results in the figures, both the OC3 and OC3-I5 cells underwent metastasis, and the entire lung in the OC3-I5 cells was filled with metastatic cells, appearing as bright red compared with the healthy part of the lung, which appear as dark red. (Figure 9) The life span of nude mice in all types of conditions (except OC3-I5) was 20 days after cancer cell implantation. By contrast, nude mice in a highly metastatic condition became sick, ate less, appeared scrawny and bony, and had difficulty moving. Irrespective of the conditions, all the nude mice had metastatic cells in the lungs; however, after shRNA knockdown of MMP-13, bright red metastatic surfaces were observed at least half of the original area. By contrast, the weight of the lungs differed; because a higher number of invasive cells were present in the lung, the lungs of the OC3-I5 cells and MMP-13-overexpression OC3 cells were heavier than those in the other conditions. These data suggested that lung metastasis might have been more severe in the MMP-13-overexpression OC3 cells than in the the OC3 cells, and that MMP-13 knockdown inhibited cancer metastasis to the lungs. However, no association was observed between metastasis and the liver. Therefore, the weight of the liver in each nude mouse was independent of the weight of the other mice. For further analysis, the lung tissue samples were trimmed, processed, embedded, and sectioned, and H & E staining was performed to examine the tissue morphologies. H & E staining of the lung revealed metastasis in the pulmonary artery and bronchial branch of the OC3-I5 cells and MMP-13-overexpression OC3 cells; metastasis in the OC3 and OC3-I5 shMMP-13-knockdown cells was rare. Overall, gross specimens and histological examination indicated that MMP-13 knockdown suppresses distant metastasis of oral cancer cells *in vivo*.

RETRACTED

**Figure 9:** Stable knockdown of MMP-13 in human oral cancer cells decreases metastasis *in vivo* (**A**) Nude mice were subcutaneously injected with OC3 and OC3-I5 cells in the tail vein. On day 20 after cancer cell implantation, the primary tumor volume was measured. On the same day, the mice were sacrificed, and the lungs were isolated and fixed in 10% formalin. The lungs were weighed. Scale bar: 2 mm. (**B**) H & E staining of OC3 and OC3-I5 and their shMMP-13-knockdown in lung metastatic tumors. Oral cancer tumor cells are indicated by the round circle with a dark purple nucleus.

## DISCUSSION

Malignant tumors have become the leading cause of death in Taiwan. In 2013, malignant tumors caused 197 deaths per 100 000 people. Among the various types of malignant tumor, tracheal, bronchus, and lung cancers remain the major causes of death [16–19]. Because the rate of tobacco smoking, alcohol abuse, and betel nut chewing are relatively high in Taiwan, oral cancer was the fifth leading cause of death (11.6 per 100 000 people). In particular, the prevalence of oral cancer is 11.9-fold higher in men than in women, and the difference in the death rate between sexes (considering other cancers) is 1.2- to 1.5-fold higher in men. After observing statistical data issued by the Ministry of Health and Welfare in Taiwan, we were motivated to study oral cancer. Tobacco smoking, excessive alcohol consumption, and betel nut chewing are the major risk factors for OSCC in Taiwan [20–22]. OSCC constitutes more than 90% of oral cancer malignancies. The 5-year survival rate of OSCC is only 50%–63% [23, 24]. In our study, we used the invasive oral cancer cell line OC3-I5, which was selected and enhanced using the transwell invasion kit more than 5 times to maintain its high penetration ability, and the parental OC3 cell line was used as the experimental line. In our previous proteomic comparison data, which were obtained using 2-dimensional difference gel electrophoresis, the 6 major factors revealing differences between the 2 cell lines were cytoskeleton composition, protein degradation, protein folding, glycolysis, redox regulation, and vesicle trafficking. The PDB name of our target protein MMP-13 is 1PEX, [25] the expression of which is 9.82-fold higher in OC3-I5 than in OC3. MMP-13 was selected because it enhances the ability of penetrating the ECM. After the cells have secreted sufficient molecules and proteins outside the cell membrane, structural and biochemical support is provided by the ECM to the surrounding cells. The ECM composition varies between multicellular structures, but cell–cell communication and differentiation are the common functions of the ECM. The ECM has numerous functions, including angiogenesis, wound repair modulation, cell cycle regulation, and niche maintenance. Collagenases (MMP-1, −8, and −13) are an abundantly secreted superfamily of MMPs, the function of which is to cleave native fibrillar type I, II, and III collagens. These 3 collagens are resistant to degradation by most proteinases and are expressed by various cell types [26–28]. Furthermore, MMP-13 accelerates the disintegration of the tight junction protein ZO-1 and hyperpermeability of the blood–brain barrier in response to hypoxia [29]. After immature part of MMP-13 has been cut, an active enzyme composed of the catalytic and hemopexin-like domains remains, and the hemopexin-like domain collaborates with other proteins to complete the collagen degradation. MMP-13 is involved in degrading the ECM during several processes such as embryonic development, reproduction, tissue remodeling, and arthritis; we focused on the effect of MMP-13 on metastasis [30]. In cancer, ECM dynamics is partly regulated by MMP superfamily to create a more favorable environment; therefore, a more advanced stage of cancer can be progressed. In ECM degradation process, MMP-13 cleaves type II collagen more efficiently than do types I and III [31, 32]. We infer that MMP-13 expression is higher in cells that are more invasive. The immunoblotting results revealed higher MMP-13 overexpression in invasive OC3-I5 cells than in the original OC3 cells; this primary phenomenon indicates that the OC3-I5 cells have high invasive ability because of the ECM degradation capability of the MMP superfamily. Moreover, MMP-13 may have been a cancer stem cell-like cell marker in several cancer cell types in previous studies [33, 34]. We obtained similar transwell invasion and migration assay results; the only difference between these 2 experiments was whether the commercial transwell was coated with Matrigel TM (BD Biosciences) in a FBS-free DMEM medium. The function of the Matrigel matrix is to mimic the ECM tissue. Using the transwell invasion assay, we examined whether the OC3 and OC3-I5 cells could degrade the matrix in the early metastatic stage. By contrast, the transwell migration assay does not coat the ECM; therefore, we sought only to determine the transformation ability of cancer cells. If cancer cells can be adequately transformed from a global shape to a sharp with more tentacles, then cancer cells easily pass through the transwell membrane. Furthermore, the transwell migration assay revealed that the migration ability of both the OC3 and OC3-I5 cells transfected with siMMP-13 significantly decreased compared with the scrambled siRNA-transfected controls (mock). After siMMP-13 knockdown, the transwell migration ability of the OC3 and OC3-I5 cells decreased by 40% and 60%, respectively. These results also indicate that MMP-13 plays a critical role in migration ability. When the primary cancer cells degrade the ECM, they can colonize anywhere in the body, particularly in organs with a high quantity of capillary blood vessels such as the lungs and kidneys. In transwell invasion and migration assays, the transwell membrane acts as a cell-membrane simulator. Aggressive cancer cells have enhanced invasion ability because of the high expression of metastasis-related proteins including MMP-13. Therefore, our approaches for inhibiting MMP-13 by using siRNA can reduce the growth and invasiveness of OC3-I5. Subsequently, siMMP-13 knockdown in the OC3-I5 cells reduced the transwell migration and invasion functions. Therefore, we observed that MMP-13 is necessary for oral cancer invasion and motility. Furthermore, Twist, Snail, and SIP are crucial in cancer metastasis [35–38]. After these proteins cooperate with each other and target a specific DNA sequence, downstream proteins, such as E-cadherin, vimentin, and the MMP superfamily, are produced [39–41]. E-cadherin is one of the most critical cellular structures and cell–matrix interaction components. E-cadherin sets cells rigidly in place; therefore, decreasing E-cadherin is considered a fundamental event in the beginning of EMT degradation. Transcription factor, such as Snail1 and Slug1, which block E-cadherin, are considered EMT-promoting factors. Slug1 binds to E-cadherin promoters and immediately represses its transcription, and Twist indirectly represses E-cadherin. This decrease in E-cadherin is accompanied with an increase in mesenchymal-associated protein expression including vimentin, N-cadherin, fibronectin, and integrin [42–45]. MMP-13-regulated cell migration involves Src signaling pathways, which induce JAM-A and vinculin expression. Moreover, Twist and SIP1 play a role in MMP-13 cell invasion. MMP-13 overexpression is higher in several tumor types (eg, breast, lung, ovary, and colon tumor tissues) than in healthy tissues. Moreover, the EMT elongation factor Snail1 is downregulated by the MMP-13–siRNA knockdown. The MMP-13 knockdown attenuates the invasive ability of oral cancer cells; p53-mediated G1 arrest was observed in MMP-13-knocked down OC3-I5 cells. Rapid migration is a characteristic of invasive cancer cells, and less E-cadherin prevents from fixed and more actin dots to elongate forward are necessary. Actin is a highly conserved cytoskeletal protein that is abundant in eukaryotic cells. High motility is characteristic of invasive cancer cells [46–48]. The cells form actin dots to attach to the ground and move forward; this phenomenon, which is called treadmilling, is crucial in cancer metastasis [49]. In cell biology, focal adhesions are large macromolecular constitutions on the surface of cells, and these assemblies can adhere to the ECM by regulating various signaling compositions, walking, and moving on the ECM [50]. Specifically, focal adhesions are the subcellular structures mediating the regulatory effects of a cell in response to ECM adhesion. Thus, the focal adhesion generates the pulling force at the adhesion site and is necessary for cells to move forward. Fluorescent microscopy revealed that MMP-13 plays a crucial role in focal adhesion formation, as indicated by the high number of actin dots; therefore, more OC3-I5 cells can attach to the culture plate compared with the OC3 and siMMP-13-knockdown cell lines. The cell cycle involves a series of stages leading to cell duplication into daughter cells. This cycle includes 4 phases (ie, G1, S, G2, and M). The cell size increases in the G1 phase, and the G1 checkpoint control mechanism ensures that conditions are feasible for DNA synthesis. During this phase, the biosynthetic activities of the cells occur at a high rate, and the increase in protein levels and the number of organelles, including the mitochondria and ribosomes, thus increase the cell size. During the G2 phase, the cells continue to grow. After the G2 checkpoint control mechanism is completed, the cells enter the M phase and divide [11–14] After siMMP-13 knockdown, both OC3 and OC3-I5 cells increase their G2/M and G1 phases, suggesting that MMP-13 downregulation induces DNA duplication and that separation is restricted until a sufficient number of energy organelles have been synthesized. Four tissue inhibitors of metalloproteinases (TIMPs) can block the catalytic domains of MMPs, and thus, the ability of remodeling the tumor microenvironment can be decreased. The EMT transcription factors Twist and calcium are key elements for regulating TIMP expression. A high level of both factors can be observed in invasive cells, which not only suppress the amount of TIMP1 mRNA, but also reduce the level of posttranslational TIMP2. Previous studies have reported that TIMP1 and TIMP2 are correlated with cancer TNM staging, and their expression is lower in metastatic cells than in nonmetastatic cells [51, 52]. Therefore, the downregulation of ECM collagens, TIMP1, and TIMP2 can be observed in invasive oral cancer cells. Inflammation can accelerate cancer initiation and progression by remodeling the tumor microenvironment. Cancer tissue inflammation can also suppress immune responses against tumor cells. Furthermore, MMPs may play the role of immune regulation in tumor microenvironments, and they may help cancer cells avoid immune surveillance. For instance, MMP-9 and -13 expression is upregulated in murine antigen, and these proteins induce arthritis and an expression pattern associated with the course of synovial inflammation. Furthermore, MMP-13 expression in mouse synovial tissues induced inflammation, and the levels of cytokine and chemokine production and inflammatory cell influx increased. MMPs are a crucial class of proteases that can alter the ECM and microenvironment. MMPs such as MMP-13 play crucial roles during the various stages of malignant tumor metastasis in tumor cell intravasation and extravasation. Some studies have also reported that MMP-13 is involved in the cancer progression of tumor cells, and others have suggested that MMP-13 has a protective role. However, the role of MMP-13 in the lung microenvironment metastasis of OSCC remains unclear. The lung is the most common metastatic site for several cancer types; therefore, it is crucial to identify molecular effectors that restrict lung metastasis. Using shRNA knockdown of MMP-13, we found that inhibiting the function of MMP-13 leads to significant decrease in lung metastasis, as evidenced by the large bright red surface area in the mock cells than in the shMMP-13-knockdown and MMP-13-overexpression cell lines. These effects suggest that MMP-13 upregulation plays a crucial role in lung metastasis. Moreover, the weight of the mice lungs differed in this study. Because more invasive cells are present in the lungs, the lungs of the OC3-I5 and MMP-13-overexpression OC3 cell lines were heavier than those of other groups. These data suggest that MMP-13-overexpression OC3 exhibited lung metastasis that was more severe than that in the OC3 cell line, and the MMP-13 knockdown inhibited tumor metastasis to the lungs. We observed a significant decrease in the tumor surface size in the MMP-13 knockdown cell lines in the lungs. However, the same phenomenon was not observed in the mice livers, suggesting that liver metastasis may occur after lung metastasis. Furthermore, if the mice were housed for a longer time, we might have observed the same phenomenon. In summary, lung metastasis occurs before liver metastasis in the metastatic cascade, and MMP-13 promotes the establishment of metastases in the liver. This observation implies that MMP-13 plays a key role in oral cancer OC3 cell metastasis. Further research must be conducted to investigate drugs that pharmacologically block metastasis in the presence of MMP-13 in humans.

RETRACTED

## MATERIALS AND METHODS

### Chemicals and reagents

Lipofectamine RNAiMAX reagent and OPTI-MEM were purchased from Life Technologies (Waltham, MA, USA); 3-(4, 5-dimethylthiazol-2-yl)-2, 5-diphenyl tetrazolium bromide (MTT) was purchased from USB Corporation (Cleveland, OH, USA); CellTiter Blue was purchased from Promega Corporation (Madison, WI, USA); SIP-1/ZEB-2, MMP-13, alpha-tubulin, Snail, Twist, and E-cadherin primary antibodies were purchased from Genetex (Hsinchu, Taiwan); phospho Src family (Tyr 416) was purchased from Cell Signaling Technology (Beverly, MA, USA); vimentin was purchased from Dako–Agilent Technologies (Glostrup, Denmark); NDE1 was purchased from AbCam (Cambridge, UK); antimouse and antirabbit secondary antibodies were purchased from GE Healthcare Sverige AB (Uppsala, Sweden); fluorescein isothiocyanate-conjugated antirabbit immunoglobulin G antibody was purchased from Jackson Immuno Research Laboratories (West Grove, PA, USA); Fetal bovine serum (FBS), trypsin–EDTA, Dulbecco modified Eagle medium (DMEM), and penicillin and streptomycin (P/S) were purchased from Gibco–Invitrogen Corporation (UK); 10-, 15-, and 4-cm Petri dishes and 96- and 24-well plates were purchased from Orange Scientific (Belgium); MTT, Tris base, glycerol, NP-40, sodium dodecyl sulfate (SDS), and tetramethylethylenediamine were purchased from USB Corporation; bovine serum albumin was purchased from Sigma–Aldrich (St. Louis, MO, USA); Horseradish peroxidase-linked antirabbit IgG was purchased from GE Healthcare BioSciences AB (Uppsala, Sweden); Tris HCl (pH 6.8) was purchased from Severn Biotech Ltd. (Kidderminster, Worcestershire, UK); HCl was purchased from Scharlau Chemie (U.S.A.); repel solution and cover oil were purchased from Amersham Pharmacia Biotech AB (Uppsala, Sweden); and an enhanced chemiluminescence substrate kit was purchased from Visual Protein Corporation. All chemicals and biochemicals used in this study were of an analytical grade.

RETRACTED

### Cell lines and cell cultures

OC3 and OC3-I5 oral cancer cells were received as a gift from Dr. Wang Lu-Hai (National Health Research Institutes, Taiwan). The OC3 cells were generated from a 57-year-old man with primary OSCC on the cheek. The OC3-I5 cells, which were OC3 cells selected from a transwell invasion assay, were reselected every 10 passages to maintain their invasive ability. Both cell lines were cultured in the DMEM medium with 10% (v/v) FBS, streptomycin (100 μg/mL), and amoxicillin and penicillin (100 IU/mL) (all purchased from Gibco–Invitrogen Corporation). The cells were maintained in a humid 5% CO_2_ atmosphere at 37°C and were passaged at 80% confluence.

### MTT cell viability assay

The cells were seeded into 96-well plates at a density of 7000 cells/well. After overnight incubation, the cells were exposed to various puromysin or G418 concentrations for 48 h; subsequently, the medium was removed and the cells were incubated in an MTT solution (1 mg/mL; 100 μL/well) at 37°C for 4 h. The supernatant was then removed, and 100 μL of dimethyl sulfoxide (DMSO) was added per well to dissolve the insoluble formazan. The 96-well plates were shaken for 10 min, and absorbance at 545 nm was measured using an ELISA reader.

### Immunoblotting assay

Immunoblotting was employed to validate the differential expression of mass spectrometry-identified proteins. The cells were lysed using a lysis buffer containing 50 mM HEPES (pH 7.4), 150 mM NaCl, 1% NP-40, 1 mM EDTA, 2 mM sodium orthovanadate, 100 μg/mL 4-benzenesulfonyl fluoride hydrochloride, 17 μg/mL aprotinin, 1 μg/mL leupeptin, 1 μg/mL pepstatin, 5 μM fenvalerate, 5 μM BpV(phen), and 1 μM okadaic acid prior to protein quantification by using a Coomassie Protein Assay Reagent (BioRad). Furthermore, 30 μg of protein samples were diluted in a Laemmli sample buffer [final concentrations: 50 mM Tris pH 6.8, 10% (v/v) glycerol, 2% SDS (w/v), and 0.01% (w/v) bromophenol blue] and separated using 1D SDS-PAGE following standard procedures. After the separated proteins were transferred onto 0.45-μm immobilon P membranes (Millipore), the membranes were blocked using 5% w/v skim milk in TBST [50 mM Tris pH 8.0, 150 mM NaCl, and 0.1% tween-20 (v/v)] for 1 h. The membranes were incubated in a primary antibody solution in TBST containing 0.02% (w/v) sodium azide for 2 h. Furthermore, the membranes were washed in TBST (3 × 10 min) and probed using the appropriate horseradish peroxidase-coupled secondary antibody (GE Healthcare). After washing in TBST 6 times (15 min each), immunoprobed proteins were visualized using an enhanced chemiluminescence substrate kit (Visual Protein Co.). All immunoblotting images were scanned using an LAS 4000 biomolecular imager (GE Healthcare, Little Chafont, UK). The antibodies used for immunoblotting are listed in the chemicals and reagents section.

RETRACTED

### siRNA design, overexpression of stable clone, and transfection

The targeting sequences 5′-GAT CTC AAG CTT ATG CAT CCA GGG GTC CA-3′ and 5′-CCA TTT TGT GGT GTC TCG AGC AGA AA-3′ against MMP-13 were designed and synthesized by Invitrogen. The sequences with similar GC content were used as the negative control against MMP-13 (Invitrogen). The OC3 and OC3-I5 cells were transfected with 60 Nm MMP-13 small interfering RNA (siRNA) or the corresponding scramble control (pGCsi) by using the Lipofectamine RNAiMAX transfection reagent (Invitrogen) according to the manufacturer's instructions. All MMP-13 cell lines were grown to 50% confluence before transfection. The Myc-DDK-tagged ORF clone of Homo sapien MMP-13 and its noncoding pCMV6-entry vector were purchased from ORIGENE–GenDiscovery Biotechnology, Inc. (New Taipei City, Taiwan). The MMP-13 cDNA was verified through sequencing. The OC3-I5 cells were also transfected with MMP-13 cDNA containing the vector or the empty vector (pcMV6) by using the Lipofectamine RNAi MAX transfection reagent (Invitrogen) according to the manufacturer's instructions. After 48 h, the AMRESCO G418 antibiotic solution (AMRESCO LLC, Solon, OH) was added at a concentration of 800 μg/mL. The population of transfectants were isolated by several subcultures and exposed to G418 for 2 months and then further examined for MMP-13 expression by immunoblotting. The OC3-I5 cells demonstrating a stable MMP-13 transfection were maintained in G418 at a concentration of 400 μg/mL, but were replaced in a complete DMEM medium for culturing at least 1 week prior to the experiment.

### Overexpression of the stable clone, lentiviral vector preparation, and infection

pLenti-IRES-Neo was purchased from ORIGENE-GenDiscovery Biotechnology, Inc., and the pLenti-MMP-13 vector was constructed by inserting MMP-13 cDNA obtained from pCMV6–MMP-13 into the empty pLenti-IRES-Neo viral vector. X-tremeGENE Transfection Reagent (Roche Diagnostics, Mannheim, Germany) was used according to the manufacturer's instructions to generate lenti–mock and lenti–MMP-13 vectors; the X-tremeGENE Transfection Reagent was diluted using the OPTI-MEM medium (Invitrogen), and plasmid DNAs (pLenti-IRES-Neo and pLenti–MMP-13) were added to the diluted X-tremeGENE reagent. The X-tremeGENE–DNA mixture was directly introduced into the HEK-293T cells. The medium was replaced after 24 h, and the supernatant, which contained lentivirus cDNA (lenti–mock and lenti–MMP-13) was collected after 72 h and filtered through 0.45-lm-pore filters. Immunoblotting was performed to evaluate the viral infection efficiency before ECC-1 infection. ECC-1 cells were transduced with lenti–mock and lenti–MMP-13 at 2 multiplicity of infection treatment levels in 2 mL of medium with polybrene (8 μg/mL) and incubated at 37°C in 5% CO_2_ for 48 h, after which the medium was replaced with a fresh DMEM culture medium.

RETRACTED

### Flow cytometry analysis for apoptosis detection and cell cycle analysis

For apoptosis detection, the percentage of apoptotic cells stained using the FITC Annexin V Apoptosis Detection kit I (BD Biosciences) was determined. The cells were trypsinized and gently washed 3 times in cold phosphate buffered saline (PBS) and then resuspended at a density of 10^6^ cells/mL in 19 Annexin V binding buffer. The cells (10^5^) were then stained with 2.5 μL of FITC-conjugated Annexin Vand 2.5 μL of propidium iodide (PI). After 20 min of incubation, the cells were analyzed using the Accuri Cflow system (BD Biosciences) by collecting emission data from the FL1 and FL2 channels at 530 and 575 m, respectively. For the cell cycle analysis, the cells were collected as described in the previous section and fixed in 1-mL of 70% ethanol overnight, followed by rehydration in 9 mL of PBS for 10 min at room temperature. The cells were then washed twice in PBS, resuspended in a PI staining solution (50 μg/mL PI stain and 100 μg/M Rnase in PBS) at a density of 10^6^ cells/mL, and incubated on ice in the dark for 30 min. The staining intensity was analyzed in 10^4^ cells by using the Accuri C6 Cflow system (BD Biosciences) to collect emission data from the FL2 channel at 575 nm. Data were further analyzed using Cflow Plus analysis software (BD Biosciences).

### Migration and invasion assay

Transwell assay was employed to examine the effect of MMP-13 on migration and invasion in MES-SA cells. Transwell cell culture inserts (PET membrane) with a pore size of 8.0 μm (SPL Life Sciences, Gyeonggi-do, Korea) were coated or not coated with Matrigel™ (BD Biosciences) in an FBS-free DMEM medium. MatrigelÔ was added to ice-cold FBS-free McCoy 5a medium at a ratio of 1:3, and 50 μL of the medium was used to coat the upper chamber of the transwell inserts. Complete medium (1 mL) was added to the lower chamber of the transwell as an attractant for the invading cells. The cells were trypsinized and washed twice in PBS, resuspended in an FBS-free McCoy 5a medium at a density of 5 × 10^5^ cells/mL, seeded in the upper chamber, and incubated at 37°C for 18 h. The noninvading cells remaining on the upper surface of the filter were removed using a cotton swab. The filters were washed 3 times in PBS, fixed in 4% paraformaldehyde for 20 min, and stained with crystal violet for 30 min. The cells that had invaded were visible under the optical microscope and were observed at a magnification of 100×.

RETRACTED

### Immunofluorescence staining

For immunofluorescence staining, MMP-13-overexpressing MES-SA cells and the relative control MES-SA cells were plated on 12-mm coverslips overnight. The cells were then fixed with 4% paraformaldehyde for 25 min, and the attached cells were washed twice in PBS, permeabilized using 0.1% Triton X100 for 10 min, and blocked with 5% bovine BSA in PBS for 1 h, followed by incubation with MMP-13 antibody (1:100) at 4°C for 24 h. After 3 washes with PBS, the samples were incubated with the appropriate fluorescent-labeled secondary antibodies (546 nm) diluted (1:100) in 2.5% BSA/PBS. For localization of the filamentous actin, the cells were incubated with 0.1 μg/mL Alexa 488–phalloidin (Sigma, St. Louis, MO, USA) for 45 min at 37°C, and the nucleus was stained with 40, 6-diamidino-2-phe-nylindole (DAPI; 1:10 000) for 1 min. The coverslips were then washed 3 times with PBS and at least twice with double distilled H_2_O before being mounted with 4-μL antifade mounting reagent (Invitrogen) and dried in the dark at 4°C. For the imaging analysis, the cells were imaged using a Zeiss Axiovert 200 M fluorescence microscope (Carl Zeiss, Jena, Germany). The same laser intensities were used for detecting identical immunostained markers, and all laser intensities used for capturing the images were not saturated. Images were exported in the TIF file format by using Zeiss Axioversion Version 4.8 and processed using Adobe Photoshop version 7.0 (Adobe Systems, San Jose, CA).

### Wound-healing migration assay

Wound-healing assay provides an easy and simple means for monitoring directional cell migration and interaction *in vitro*. We seeded 2 × 10^5^ OC3 and OC3-I5 cells with or without siRNA treatment into 12-well dishes and incubated them for 24 h (approximately 90% confluence). A linear wound was generated by passing a sterile 10-μL plastic pipette tip through a premarked line. After the cells were washed 3 times with PBS to remove serum and cell debris, they were incubated in a serum-free medium for 24 h at 37°C in 5% CO_2_. The wound of each condition was photographed at 0, 8, 16, and 24 h immediately above the intersection of the wound areas and premarked lines. The wound areas were calculated using AxioVision version 4.

RETRACTED

### MTT cell viability assay

The cells were seeded into a 96-well dish at a density of 8000 cells/well. After 48 h, the medium was removed and the cells were incubated in an MTT solution (1 mg/mL; 100 μL/well) at 37°C for 4 h. After removing the supernatant, 100 μL of DMSO was added to each well to dissolve the insoluble formazan. The 96-well dish was then shaken for 10 min, and the absorbance at 545 nm was measured using an ELISA reader.

### Orthotopic tumor implantation

Five-week-old BALB/cAnN.Cg-Foxnlnu/CrlNarl female mice were housed in a specific-pathogen-free environment. After being house for 1 week, the mice were injected with human oral cancer cells. Furthermore, the mice received an intravenous injection of 2 × 10^6^ OC3 and OC3-I5 cells (with or without shMMP-13 knockdown cell lines) mixed with 100 μL of 1X PBS. The cells were subcutaneously inoculated into a vein in the tail of the mice after stimulating the dilation of the tail veins by placing the mice under an infrared light source in a warmer environment (e.g. (48°C–55°C) for 1 min (6 per group). The mice were sacrificed using zoletil/rompun 3 weeks after implantation, and the lungs were removed and fixed in 10% formalin. For further analysis, the lung tissue samples were trimmed, processed, embedded, sectioned, and subjected to hematoxylin and eosin (H & E) staining to examine the tissue morphologies. These procedures were performed by the National Laboratory Animal Center, Taiwan, R.O.C. All the mice were fed ad libitum and housed in accordance with the guidelines of the Society of Laboratory Animal Science.

### Statistical analysis

The Student *t* test and analysis of variance were employed for the statistical analysis, with *P* < .05 considered statistically significant.
